# Bayesian Estimation of Different Scale Parameters Using a LINEX Loss Function

**DOI:** 10.1155/2022/4822212

**Published:** 2022-04-30

**Authors:** M. A. Mohammed, Sundus N. Al-Aziz, Eateraf M. A. Al Sumati, Emad E. Mahmoud

**Affiliations:** ^1^Department of Mathematics, Al-Lith University College, Umm Al-Qura University, Mecca, Saudi Arabia; ^2^Department of Mathematics, Faculty of Science, Assiut University, Assiut, Egypt; ^3^Department of Mathematical Sciences, College of Science, Princess Nourah bint Abdulrahman University, P.O. Box 84428, Riyadh 11671, Saudi Arabia; ^4^Department of Statistics & Informatics, Faculty of Administrative Sciences, University of Aden, Aden, Yemen; ^5^Department of Mathematics and Statistics, College of Science, Taif University, P.O. Box 11099, Taif 21944, Saudi Arabia

## Abstract

The LINEX loss function, which climbs exponentially with one-half of zero and virtually linearly on either side of zero, is employed to analyze parameter analysis and prediction problems. It can be used to solve both underestimation and overestimation issues. This paper explained the Bayesian estimation of mean, Gamma distribution, and Poisson process. First, an improved estimator for *μ*^2^ is provided (which employs a variation coefficient). Under the LINEX loss function, a better estimator for the square root of the median is also derived, and an enhanced estimation for the average mean in such a negatively exponential function. Second, giving a gamma distribution as a prior and a likelihood function as posterior yields a gamma distribution. The LINEX method can be used to estimate an estimator $\hat{\lambda_{BL}}$ using posterior distribution. After obtaining $\hat{\lambda_{BL}}$, the hazard function $\hat{h_{BL}}$ and $\hat{D_{BL}}$ the function of survival estimators are used. Third, the challenge of sequentially predicting the intensity variable of a uniform Poisson process with a linear exponentially (LINEX) loss function and a constant cost of production time is investigated using a Bayesian model. The APO rule is offered as an approximation pointwise optimal rule. LINEX is the loss function used. A variety of prior distributions have already been studied, and Bayesian estimation methods have been evaluated against squared error loss function estimation methods. Finally, compare the results of Maximum Likelihood Estimation (MLE) and LINEX estimation to determine which technique is appropriate for such information by identifying the lowest Mean Square Error (MSE). The displaced estimation method under the LINEX loss function was also examined in this research, and an improved estimation was proposed.

## 1. Introduction

The LINEX loss function is a nonlinear function that climbs exponentially with one end of 0 and virtually exponentially on another [1]. For values approaching zero, this error function reduces to squared error loss. For calculating the binomial variable, the LINEX loss function is used. This loss function was used to estimate the median of a normally distributed [2]. Consider the prediction error in the perspective of exponential distribution reliability analysis. Then, using the LINEX loss function, Bayesian mean and square mean estimations of a normally distributed were investigated. Under the LINEX loss function, the MMSE criterion is unacceptable. The uniformly minimum risk unbiased (UMRU) estimator under the LINEX loss function can be found using information and facts if there is underestimation and overestimation in real-life situations [3]. The exponential distribution is a well-known distribution that may be used in a variety of fields, including science, economy, and demographics [4]. It is a well-known one-parameter distribution that is frequently utilized in model studies [5].

A linear exponential loss function (LINEX) is developed to estimate the scale parameter and reliability function of the inverse Weibull distribution (IWD) based on lower record values [6]. The Bayesian technique is also necessary for this study, in addition to employing Maximum Likelihood to estimate the parameters. It creates a posterior probability by combining an exponential distribution's likelihood value with a prior [7]. Because altering the value to 1 and having an Exponential distribution, the Gamma distribution is an appropriate prior for it. In statistics, there are a few estimating approaches. One of them is Bayesian, which finds the posterior distribution using the likelihood function and prior distribution [8]. The data is exponentially distributed, and the posterior distribution will be constructed using a Gamma distribution as its prior. Let *F* be sometimes referred to as the failure time random variable because it is defined as the time of failure of the object known to exist at time *t* = 0. If *F* is the time to failure, the likelihood of still operating at time *t*  is like the probability that the failure will occur later (mathematical model higher) than *t*. The following equation is the definition of the survival density function (SDF), probability density function (PDF), and hazard rate function (HRF).

(1) $$\begin{array}{c} D\left(t\right)=e^{-\lambda t},t\geq 0.\;\lambda \geq 0,\\ p\left(t\right)=-\frac{d}{dt}D\left(t\right)=\lambda e^{-\lambda t},\\ \lambda \left(t\right)=\frac{p\left(t\right)}{D\left(t\right)}=\lambda . \end{array}$$

The task of establishing appropriate halting rules is frequently and analytically intractable. Because determining explicit optimum ending times is challenging, numerous approaches were proposed to obtain “asymptotically” optimal regulations [9]. For example, it offered simple but appealing large enough sample approximations to optimal timings, dubbed asymptotically pointwise optimal (APO) rules, and demonstrated that APO rules were asymptotically optimal (AO) under a second scenario. Many publications have examined the APO rule and how it might be used to address those other challenges [10]. Discrete-time events are the focus of the studies in these publications. They discussed how the LINEX error function operated, but still, no specifics or practical solutions were provided on how the LINEX loss function changes the shape variable and error value [11]. Considering the LINEX loss method's versatility in estimating a location parameter, it does not seem to be useful for estimating scale variables and other values. For two variables, Bayes and probability estimators are used [12]. Under hazard and survival variables used in experiments and analysis methods, Weibull using unfiltered observations is examined.

In continuous-time processes, the idea of the asymptotic element-wise optimization problem is expanded from discrete-time processes [11]. Additionally, with a squared error loss, the APO procedures for predicting the intensities of a homogeneity Poisson process are AO for random priors and asymptotically nondeficient for conjugation priors [13]. Later, it generalized a conclusion for continuous-time processes and demonstrated that under a linear exponential (LINEX) loss function, the APO rules for such a Poisson distribution are AO for such corresponding priors [14]. The LINEX loss function was officially created, and its properties were investigated further. It is a handy asymmetrical nonlinear function that increases dramatically on one end of zero and gradually on the other [15]. Much research has looked into estimating issues with LINEX loss function [16]. After analyzing the data, it assigns relative weights to each given value. Approximations to Bayesian inference exist, such as the Specific Noninformative Prior [17]. Linear Exponential Loss Function, Lindley Approximation, General Entropy Loss Function, and Squared Error Loss Function are all examples of linear, exponential loss functions.

## 2. Related Work

The Weibull distribution is commonly used in lifespan data modeling and analysis [14]. The considered wide range of a two-parameter Weibull distribution having given shape is estimated in this study. How to use estimated parameters is discussed. Under the LINEX loss function, the Bayes estimator is produced utilizing Jeffreys' prior. Using generated data sets, the overall performance of the estimation techniques is calculated in small and large sampling for overestimation and underestimation. It has been discovered that the Bayes estimator performed best in observational studies and then when overstatement is much more important than underestimating.

In technology, science, and other fields, the Weibull distribution has been identified as among the most effective distributions for predicting and evaluating lifetime data [18]. To find the most effective approach for calculating its characteristics, the Bayesian estimate strategy for estimation methods, which competes with other estimation approaches, has suddenly received a lot of attention. For assessing the 2 different Weibull failure time distributions, the achievement of the maximum likelihood method and Bayes estimator using expansions of Jeffreys prior knowledge with three wavelet coefficients, namely, the sequential exponential loss, general electron density loss, and square error linear function. Through a simulation analysis with varied sample sizes, these approaches are evaluated using mean square error. The findings demonstrate that for certain values of extensions of Jeffreys' prior, the Bayesian estimator utilizing extensions of Jeffreys' prior with linear exponentially error function has the minimum mean square error and actual bias both for weighting factor and the significant impact.

Dey introduced Bayes' estimation technique for such an Inverse Rayleigh distribution's unknown quantity (IRD) [19]. Utilizing noninformative prior, Bayes estimation techniques are derived for symmetrical (squared error (SE) loss) and asymmetrical linear exponential loss functions. The estimators' system is assessed based on its relative hazard under two wavelet coefficients. They also construct the reliability method's Bayesian estimation method using symmetrical and asymmetrical loss functions and compare their efficiency that used a Monte Carlo simulation analysis. Lastly, to highlight the findings, a numerical investigation is offered.

Gupta presented a new method for predicting the variable of the Rayleigh distribution, Bayesian and E–Bayesian estimate methods are provided in this study [20]. The parameter's Bayes estimation is calculated using the LINEX loss function and the concept that the prior probability is relevant, i.e., gamma distribution. Furthermore, a simulation study utilizing MATLAB software was used to compare the E-Bayes estimation method with related Bayes estimators.

The work of Lee and Hwang looks at the challenge of progressively predicting the average of a Poisson process in a Bayesian network using a LINEX (linear exponential) loss function and a fixed price per experience [21]. For arbitrary priors, an approximation pointwise optimum rule with such a distribution function is developed and proven to be exponential optimal. An actual data set is used to demonstrate the suggested monotonically elementwise optimum rule.

## 3. Proposed Methodology

Let us consider *a*_1_, *a*_2_,……*a*_*n*_ an n-person representative sample from such an average distribution with median *μ* and variance *σ*^2^. Assume that compared to the population median with minimum error $\bar{a}=\left(\sum^{}a_{i}/n\right)$, the sample mean (*σ*^2^/*n*) is an adequate and accurate estimator. The standard approach of comparing estimation methods for the significant feature using mean square error (MSE) may not provide a clear favorite for scale parameters [22]. Limiting the class of estimators is one technique to make the task of finding the “best estimator” more tractable. Consider impartial and partially invariant estimation techniques as a popular approach to limiting the category of estimation techniques.

The improvement of the estimator $E^{\prime }=\left(n\bar{a}/n+v^{2}\right)$is in the estimator class $E^{\prime }=s\bar{a}$ and it shows the MSE represented in the equation:

(2) $$\begin{array}{c} \text{MSE}\left(E^{\prime }\right)=\frac{\sigma^{2}}{n}{\left(1+\frac{\sigma^{2}}{n}\right)}^{-1}<MSE\left(\bar{a}\right)=\frac{\sigma^{2}}{n}. \end{array}$$

*U*(*a*)=*θ*,  *R*(*a*)=*θ*^2^ and *v*=1 in the negative exponential distribution (NED). The scale parameter is *θ*, and the improved estimator is $E_{1}=\left(n\bar{a}/n+1\right)$ with an MSE *E*_1_=(*θ*^2^/*n*+1) lower than (*θ*^2^/*n*). In a normal distribution with mean *μ* and variance *σ*^2^, where *σ*^2^ acts as a standard deviation and the maximum likelihood estimate are $M^{2}=\left(1/n\right)\sum^{}{\left(a_{1}-\bar{a}\right)}^{2}$ (MLE), the estimators for *σ*^2^ (the unbiased estimator).

Thus, MSE (*M*^2^)=(2*σ*^4^/*n*) and then MSE. (*M*^2^)=(2*σ*^4^/*n* − 1)

The LINEX loss equation is given below:

(3) $$\begin{array}{c} L\left(\Delta ,x\right)=y\left[e^{x\Delta }-x\Delta -1\right],\;\Delta =\hat{\mu }-\mu ,\;x\neq 0, \end{array}$$

where *x* and *y* are the shapes and a scale parameter.

If |*x*|⟶0, Square inaccuracy is the result of the LINEX loss.

Mean Estimation using a LINEX loss function.

$L\left(x,\Delta \right)=y\left(e^{x\Delta }-z\Delta -1\right),\;\Delta =\hat{\mu }-\mu ,$ *x* ≠ 0, and if the *bc*=*x*,   Later, this procedure would equal *y*(*e*^*x*Δ^ − *z*Δ − 1)

The loss function of LINEX minimizes the squared error if *|x|*⟶0.

For calculating, the constant form of LINEX loss was used. LINEX loss in its symmetric form is given in the equation:

(4) $$\begin{array}{c} L\left(x,\Delta^{*}\right)=y\left(e^{x\Delta^{*}}-z\Delta^{*}-1\right),\Delta^{*}=\frac{\hat{\mu }}{\mu }-1,\;x\neq 0,\\ Q\left(x,\Delta^{*}\right)=W\left[L\left(x,\Delta^{*}\right)\right]=\frac{x^{2}}{2}\left[W\left({\left.\frac{z\bar{a}}{\mu }-1\right)}^{2}\right.+\frac{x}{3}W\left({\left.\frac{z\bar{a}}{\mu }-1\right)}^{3}+\ldots \right.\right], \end{array}$$

where $\hat{\mu }=z\bar{a}$

$\left(2/x^{2}\right)Q\left(x,\Delta^{*}\right)=W\left[\left({\left.\bar{a}/\mu -1\right)}^{2}\right.\right]+\left(x/3\right)W\left[\left({\left.z\bar{a}/\mu -1\right)}^{3}\right.\right]+\ldots$

Consider the estimator *Y* = xc 1 in the case of a normally distributed with variance and mean both equal to two. LINEX loss in its invariant form is given in the following equation:

(5) $$\begin{array}{c} L\left(x,\Delta^{*}\right)=e^{x\left(\left(z\bar{a}/\mu \right)-1\right)}-x\left(\frac{z\bar{a}}{\mu }-1\right)-1,\\ Q\left(x,\Delta^{*}\right)=e^{x^{2}z^{2}v^{2}/2n}e^{-x\left(1-z\right)}-xz+x-1,\\ \frac{2}{x^{2}}Q\left(x,\Delta^{*}\right)=\frac{xz^{3}}{3}\left(1+\frac{3v^{2}}{n}\right)e^{-x}+\frac{z^{2}}{2}\left(1+\frac{v^{2}}{n}\right)e^{-x}-\left(2-x+\frac{x^{2}}{3}-\frac{x^{3}}{12}\right)+1-\frac{x}{3}+\frac{x^{2}}{12}. \end{array}$$

In a negative exponential distribution,

(6) $$\begin{array}{c} E\left[e^{xz\bar{a}/\theta }\right]=\left({\left.1-\frac{xz}{n}\right)}^{-n}\right.\;,\\ Q\left(x,\Delta^{*}\right)=\frac{e^{-x}}{\left({\left.1-\left(xz/n\right)\right)}^{n}\right.}-xz+x-1. \end{array}$$

From equation (8), then the value of minimum *z* could be shown in the following equation:

(7) $$\begin{array}{c} z_{\text{min}}=\frac{n}{x}\left(1-e^{-\left(x/\left(n+1\right)\right)}\right). \end{array}$$

The proposed estimation is $E_{1}=\left(n/x\right)\left(1-e^{\left(-x/n+1\right)}\right)\bar{a}$ with a. Min*Q*(*x*, Δ^*∗*^)=*x* − (*n*+1)(*x* − *e*^(−*x*/*n*+1)^)

As a result, under the LINEX loss function, the minimum mean squared error is unacceptable [7]. This can get the minimum if the differentiate equation (5) is about *c* and equal to zero:

(8) $$\begin{array}{c} z_{\text{min}}=\left[\frac{\left(x-1\right)\left(1+\left(v^{2}/n\right)\right)+\sqrt{{\left(1-x\right)}^{2}\left({\left.1+\left(v^{2}/n\right)\right)}^{2}+4\left(x-\left(x^{2}/2\right)\right)\left(1+\left(3v^{2}/n\right)\right)\right.}}{a\left(1+\left(3v^{2}/n\right)\right)}\right]\;. \end{array}$$

The values of *z* can be calculated given the values of *n*,  *v* ≥ 1 and 0 ≤ *x* ≤ 0.6. Then, get the lowest risk by plugging the *c*_min_ into equation (5) [23]. Figures 1–3 show the relative effectiveness of the estimator *E*_1_ in comparison to *E*′ for *v*=2.00(2.25)2.50,  *x*=0.2(0.4)0.6  and *n* = 5(5)20. The figure illustrates that if *v* ≥ 1  is greater than 1, the estimator outperforms with smaller *n* values and a level up to 2.00.

Also, under the LINEX loss function, the Bayesian estimator for median and square of group means of normally distributed was investigated. In the case of a negative exponential function, the answer for the scale parameter by using an invariant form of the LINEX error function is $E_{1}=\left(n/x\right)\left(1-e^{\left(-x/n+1\right)}\right)\bar{a}$

(9) $$\begin{array}{c} E_{1}=\frac{n\bar{a}}{n+1}-\frac{xn\bar{a}}{2{\left(n+1\right)}^{2}}+\frac{xn\bar{a}}{6{\left(n+1\right)}^{3}}\ldots \end{array}$$

$\left(2n\bar{a}/\theta \right)$ (Gamma (1, *n*)) adopts a chi-square distribution with 2*n* degrees of freedom. It established a modified Bessel formula as follows:

(10) $$\begin{array}{c} B_{n}\left(2nx\bar{a}\right)=1+\frac{2nx\bar{a}}{1!n}+\frac{4x^{2}n^{2}\bar{a^{2}}}{2!n\left(n+1\right)}+\frac{8x^{3}n^{3}\bar{a^{3}}}{2!n\left(n+1\right)\left(n+2\right)}+\ldots \\ =1+2x\bar{a}+\frac{4x^{2}n\bar{a^{2}}}{2\left(n+1\right)}+\ldots \\ E\left[E_{n}\left(2nx\bar{a}\right)\right]=1+2x\theta +\frac{x^{2}}{2!}4\theta^{2}+\ldots \;=e^{2x\theta }\\ \log\;E\left[E_{n}\left(2nx\bar{a}\right)\right]=2x\theta ⟶\frac{1}{2x}\log\;E\left[E_{n}\left(2nx\bar{a}\right)\right]=\theta . \end{array}$$

The estimator MVRU for *θ* is as follows:

(11) $$\begin{array}{c} \hat{\theta }=\bar{a}-\frac{x\bar{a^{2}}}{\left(n+1\right)}+\ldots \end{array}$$

This demonstrates that in the LINEX loss function, adequate statistics *x* can also be used to determine the UMRU estimation.

### 3.1. Maximum Likelihood Estimation

Censoring is a method of dealing with incomplete data that occurs as a result of events such as death, loss, or removal from observation. Variables *V*_1_,…*V*_*n*_ denote *n* individual lifespan, as per [24]. A lifetime or a counting time is denoted by the letter *v*_*i*_. The censoring or state indication for *t*_1_ is the variable *δ*_*i*_=1 if *V*_*i*_=*t*_*i*_ and 0 if *V*_*i*_  >  *t*_*i*_. The value t1 is calculated using min(*V*_*i*_,  *Z*_*i*_),  *i*= 1,2,3, ...,  *n*, where *V*_*i*_ is the length of their remission assessed from the beginning of the course and *Z*_*i*_ is the period between the beginning of the study and the end of the study. It is possible to construct the likelihood function of censored data for observations (*t*_*i*_, *δ*_*i*_)*i*=1,2, ...,  *n*.

(12) $$\begin{array}{c} K\left(t_{i};\delta ,\lambda \right)=\overset{n}{\underset{i=1}{\prod }}{\left[f\left(t_{1};\lambda \right)\right]}^{\delta_{i}}{\left[R\left(t_{i};\lambda \right)\right]}^{1-\delta_{i}}. \end{array}$$

The exponential distribution likelihood function for the observation (*t*_*i*_, *δ*_*i*_)*i*=1,2,3,…, *n* is calculated as follows:

(13) Kti;δ,λ=∏i=1nλe−λtiδiRe−λti1−δi=λδ1,λδ2,…,λδne−λt1,e−λt2,…,e−λtn=λ∑i=1nδie−λ∑i=1nti

Then, as shown above, discover a natural logarithm of the likelihood function.

(14) $$\begin{array}{c} k=\ln\;K\left(t_{i};\lambda ,\delta \right)=\left(\overset{n}{\underset{i=1}{\sum }}\delta_{i}\right)\ln\;\lambda -\left(\overset{n}{\underset{i=1}{\sum }}t_{i}\right)\lambda . \end{array}$$

By deriving *k* to the parameter *λ*,  , obtain the following:

(15) $$\begin{array}{c} \frac{dk}{d\lambda }=0,\\ \frac{d}{d\lambda }\left[\left(\overset{n}{\underset{i=1}{\sum }}\delta_{i}\right)\ln\;\lambda -\left(\overset{n}{\underset{i=1}{\sum }}t_{i}\right)\lambda \right]=0,\\ \frac{\sum_{i=1}^{n}\delta_{i}}{\lambda }-\overset{n}{\underset{i=1}{\sum }}t_{i}=0,\\ \lambda =\frac{\sum_{i=1}^{n}\delta_{i}}{\sum_{i=1}^{n}t_{i}}. \end{array}$$

A Maximum Likelihood Estimated is obtained. Subsequently, both the equation of survival and the rate of hazard are composed.

(16) $$\begin{array}{c} \hat{D_{ML}}\left(t_{i};\hat{\lambda }\right)=e^{-\hat{\lambda }t_{i}}=e^{-\left(\overset{n}{\underset{i=1}{\sum }}\delta_{i}/\overset{n}{\underset{i=1}{\sum }}t_{i}\right)t_{i}},\\ \hat{E_{ML}}\left(t_{i};\hat{\lambda }\right)=\hat{\lambda }=\frac{\sum_{i=1}^{n}\delta_{i}}{\sum_{i=1}^{n}t_{i}}. \end{array}$$

$\hat{D_{ML}}\left(t_{i};\hat{\lambda }\right)$ and $\hat{E_{ML}}\left(t_{i};\hat{\lambda }\right)$ are based on Maximum Probability [2]. The ratio of hazard and survival model is estimated.

### 3.2. The Poisson Process Rules of APO and AO

Let {*N*(*f*) : *f* ≥ 0} be a Poisson process that is homogeneous but has an undetermined amplitude parameter. It is desired to predict *θ* by $\tilde{\theta_{f}}=\tilde{\theta_{f}}\left(N\left(s\right):0\leq s\leq f\right)$, a specific topic to the LINEX loss and the sampling cost after observing the process during the time interval [0,  *f*].

(17) $$\begin{array}{c} K\left(\tilde{\theta_{f}},\theta \right)+zf, \end{array}$$

where $K\left(\theta ,\tilde{\theta_{f}}\right)=\exp\left[x\left(\tilde{\theta_{f}}-\theta \right)\right]-x\left(\tilde{\theta_{f}}-\theta \right)-1,\;x\neq 0,$ is the price per unit time, *c* is the LINEX loss. As can be seen, *c* can also be thought of as a proportional weight to the LINEX loss. Across all stopping periods and estimation methods, the goal is to minimize the Bayes hazard. Concerning the defect $\tilde{\theta_{f}}-\theta$, the LINEX loss is a positive and asymmetrical function [25]. It is beneficial in estimating difficulties when underestimation or overestimation is deemed more dangerous than the other. The shape of the object is determined by the variable a. When the *x* > 0, it means that overestimation is more expensive than underestimation. When *x* < 0 is present, the inverse is true.

Assume, which has a *θ* constant density Ψ concerning the Lebesgue measurement, with *L*(*θ*) < *∞* and *L*(*e*^−*xθ*^) < *∞*, respectively. For ℱ_'_=*σ*(*N*(*u*) : 0 ≤ *u* ≤ *f*) for *f* ≥ 0 and ℱ_*∞*_ be the smallest -field comprising all of ℱ_'_ events for all *f* ≥ 0. The Bayesian estimation is very well recognized as the best estimation with a stop time of P.

(18) $$\begin{array}{c} \tilde{\theta_{p}}=-\frac{1}{x}\log\;L\left(e^{-x\theta }|{ℱ}_{p}\right), \end{array}$$

where ℱ_*p*_={*X* ∈ ℱ_*∞*_|*X*|∩{*N* ≤ *f*} ∈ ℱ_*f*_ forall *f* ≥ 0}. The Bayes hazard of a Bayesian sequential approach $\left(N,\;\tilde{\theta_{N}}\right)$ is therefore equal to the following:

(19) $$\begin{array}{c} E\left[xE\left(\theta |{ℱ}_{N}\right)+\log\;E\left(e^{-x\theta }|{ℱ}_{N}\right)+zN\right]\;, \end{array}$$

This suggests an APO condition in a Poisson distribution as in Section 3.2.

*τ*_*z*_^*∗*^=inf{*f* ≥ 0 : *xE*(*θ|*ℱ_1_)+log  *E*(*e*^−*xθ*^*|*ℱ_1_) ≤ *zf*}, *z* > 0.

In Theorem 1, the halting rule *τ*_*z*_^*∗*^ and the Bayesian sequential process $\left(\tau_{z}^{*},\tilde{\theta_{\tau_{z}^{*}}}\right)$ are proven to be APO and AO, respectively. To establish Theorem 1, first establish some representations, followed by the development of some supplementary results. Let $\hat{\theta_{f}}=\left(W\left(f\right)/f\right)$ be the maximum likelihood estimation *θ* of based on {*W*(*i*) : 0 ≤ *i* ≤ *f*}, and define Ψ^*∗*^(*a|*ℱ_*f*_) as the posterior probability of $\sqrt{f}\left(\theta -\hat{\theta_{f}}\right)$ given ℱ_*f*_ for simplicity. Thus,

(20) $$\begin{array}{c} \Psi^{*}\left(a|{ℱ}_{f}\right)=\frac{{\left(\hat{\theta_{f}}+a/\sqrt{f}\right)}^{W\left(f\right)}e^{-\left(\hat{\theta_{f}}+\left(a/\sqrt{f}\right)\right)f}\Psi \left(\hat{\theta_{f}}+\left(a/\sqrt{f}\right)\right)}{\sqrt{f}\int_{0}^{\infty }N^{W\left(f\right)}e^{-Nf}\Psi \left(N\right)dn},a>-\hat{\theta_{f}}\sqrt{f}. \end{array}$$

Define the random numbers

(21) $$\begin{array}{c} R_{t}\left(a\right)=\text{exp}\left\{\left[W\left(f\right)\ln\left(\hat{\theta_{f}}+\frac{a}{\sqrt{f}}\right)-\left(\hat{\theta_{f}}+\frac{a}{\sqrt{f}}\right)f\right]-\left[W\left(f\right)\ln\hat{\theta_{f}}-\hat{\theta_{f}}f\right]\right\}. \end{array}$$

For $a>-\hat{\theta_{f}}\sqrt{f}$ and *B*_*f*_(*a*)=0 otherwise, then

(22) $$\begin{array}{c} Q_{t}\left(b\right)=\frac{1}{f}\left\{\left[W\left(t\right)\ln\left(\hat{\theta_{f}}|+|b\right)-\left(\hat{\theta_{f}}+b\right)f\right]-\left[W\left(f\right)\ln\hat{\theta_{f}}-\hat{\theta_{f}}f\right]\right\}. \end{array}$$

For $b>-\hat{\theta_{f}}$ and *Q*_*t*_(*b*)=−1.

### 3.3. The LINEX Loss Function of Bayesian

In statistical methods studies, the Bayesian Process is the well-estimating method [26]. The Bayesian estimate has three different loss functions. In Bayesian estimation, another of the loss functions is LINEX. As per Zellner, the LINEX loss method's posterior prediction [27]. One of the Bayesian techniques is the LINEX loss function. The variable estimation of *λ* is represented by ${\hat{\lambda }}_{lin}$ that under LINEX error function is constructed while using Zellner's method.

(23) $$\begin{array}{c} {\hat{\lambda }}_{lin}=-\frac{1}{z}\ln\left[E\left(e^{-z\lambda }\right)\right]. \end{array}$$

To expose the posterior equation which can be utilized to find a parameter estimate BL under the Bayesian LINEX loss function.

(24) $$\begin{array}{c} E\left(e^{-z\lambda }\right)=\overset{\infty }{\underset{0}{\int }}e^{-z\lambda }p\left(\lambda |t_{i}\right)d\lambda \;,\\ =\overset{\infty }{\underset{0}{\int }}e^{-z\lambda }\left[\frac{\left({\left.\sum_{i=1}^{n}t_{i}+\beta \right)}^{\sum_{i=1}^{n}\delta_{i}+\alpha }\lambda^{\sum_{i=1}^{n}\delta_{i}+\alpha -1}e^{-\lambda \left(\sum_{i=1}^{n}t_{i}+\beta \right)}\right.}{\Gamma \left(\sum_{i=1}^{n}\delta_{i}+\alpha \right)}\right]d\lambda ,\\ =\frac{{\left(\sum_{i=1}^{n}t_{i}+\beta \right)}^{\sum_{i=1}^{n}\delta_{i}+\alpha }\Gamma \left(\sum_{i=1}^{n}\delta_{i}+\alpha \right)}{{\left(\sum_{i=1}^{n}t_{i}+\beta +z\right)}^{\sum_{i=1}^{n}\delta_{i}+\alpha }\Gamma \left(\sum_{i=1}^{n}\delta_{i}+\alpha \right)},\;\\ =\left({\frac{\sum_{i=1}^{n}t_{i}+\beta }{\sum_{i=1}^{n}t_{i}+\beta +z}}^{\overset{n}{\underset{i=1}{\sum }}\delta_{i}+\alpha }\right), \end{array}$$

As a result of (24) get the appropriate estimation method under the LINEX loss function:

(25) $$\begin{array}{c} {\hat{\lambda }}_{BL}=-\frac{1}{z}\ln\left[E\left(e^{-z\lambda }\right)\right],\\ =-\frac{1}{z}\ln\left[\left({\left.\frac{\sum_{i=1}^{n}t_{i}+\beta }{\sum_{i=1}^{n}t_{i}+\beta +z}\right)}^{\sum_{i=1}^{n}\delta_{i}+\alpha }\right.\right], \end{array}$$

Furthermore, equation (26) describes the survival and hazard functions [16] that under a LINEX loss function,

(26) $$\begin{array}{c} \hat{D_{ML}}\left(t_{i};\hat{\lambda }\right)=e^{-\hat{\lambda }t_{i}},\\ =e^{-\left(\frac{1}{z}\ln\left[\left({\left.\frac{\sum_{i=1}^{n}t_{i}+\beta }{\sum_{i=1}^{n}t_{i}+\beta +z}\right)}^{\sum_{i=1}^{n}\delta_{i}+\alpha }\right.\right]\right)t_{i}},\\ \hat{E_{ML}}\left(t_{i};\hat{\lambda }\right)=\hat{\lambda },\\ =-\frac{1}{z}\ln\left[\left({\left.\frac{\sum_{i=1}^{n}t_{i}+\beta }{\sum_{i=1}^{n}t_{i}+\beta +z}\right)}^{\sum_{i=1}^{n}\delta_{i}+\alpha }\right.\right]\;. \end{array}$$

### 3.4. Square Estimation of Mean by Using LINEX Loss Function

In the normal distribution, thus known as follows:

(27) $$\begin{array}{c} N\left(\bar{a}\right)=\frac{\sigma^{2}}{n}. \end{array}$$

That implies the following:

(28) $$\begin{array}{c} {\hat{\mu }}^{2}=\frac{{\bar{a}}^{2}}{1+\left(v^{2}/n\right)}, \end{array}$$

Let us consider the minimum value of *t*_2_

(29) $$\begin{array}{c} U_{2}=t_{2}{\bar{a}}^{2},\\ t_{2\text{min}}=\frac{1+\left(v^{2}/n\right)}{\left({\left.1+\left(v^{2}/n\right)\right)}^{2}+v^{2}/n\left(4+\left(v^{2}/n\right)v^{2}\right)\right.}\leq 1. \end{array}$$

Then the estimator proposed is represented as follows:

(30) $$\begin{array}{c} U_{2}=\frac{{\bar{a}}^{2}}{1+\left(v^{2}/n\right)\left\{1+\left(4+\left(v^{2}/n\right)/1+\left(v^{2}/n\right)\right)\right\}}. \end{array}$$

If *v* is known (30); if *v* is unknown; then MVUE for *μ*^2^ is as follows:

(31) $$\begin{array}{c} N={\bar{a}}^{2}-\frac{d^{2}}{n}. \end{array}$$

*N* could be negative for smaller values of *n*, hence proposed a biassed estimator for *μ*^2^ as $S=\left({\left.1+\left(d^{2}/n{\bar{u}}^{2}\right)\right)}^{-1}{\bar{a}}^{2}\right.$ and looked at its huge sample features [28]. To generate an estimator with a certain mean square error as *S* but a reduced bias than *S* for huge sample sizes *n*,

(32) $$\begin{array}{c} K=\frac{{\bar{a}}^{2}}{1+\left(d^{2}/n{\bar{u}}^{2}\right)\left[1+\left(d^{2}/n{\bar{u}}^{2}\right)\right]}. \end{array}$$

For the estimator, the invariant expression of the LINEX loss function

(33) $$\begin{array}{c} U_{4}=t_{4}{\bar{a}}^{2}\\ L\left(x,\Delta^{*}\right)=e^{-x}e^{x{\bar{a}}^{2}t_{4}/\mu^{2}}-x\left(\frac{x{\bar{a}}^{2}t_{4}}{\mu^{2}}-1\right)-1,\\ Q\left(x,\Delta^{*}\right)=e^{-x}W\left[e^{x{\bar{a}}^{2}t_{4}/\mu^{2}}\right]-xW\left[\frac{x{\bar{a}}^{2}t_{4}}{\mu^{2}}-1\right]-1,\\ \frac{2}{x^{2}}Q\left(x,\Delta^{*}\right)=\frac{xt_{4}^{3}}{3}W\left(\frac{{\bar{a}}^{6}}{\mu^{6}}\right)e^{-x}+\frac{t_{4}^{2}}{2}W\left(\frac{{\bar{a}}^{4}}{\mu^{4}}\right)e^{-x}-\left(2-x+\frac{x^{2}}{3}-\frac{x^{3}}{12}\right)\left(1+\frac{v^{2}}{n}\right)t_{4}+1-\frac{x}{3}+\frac{x^{2}}{12}. \end{array}$$

This gets to *t*_4_ and equal to zero by simplifying this solution.

(34) $$\begin{array}{c} t_{4m}=\frac{-W\left({\bar{a}}^{4}/\mu^{4}\right)+\sqrt{W^{2}\left({\bar{a}}^{4}/\mu^{4}\right)}+e^{x}\left(2-x+\left(x^{2}/3\right)-\left(x^{3}/12\right)\right)\left(1+\left(v^{2}/n\right)\right)W\left({\bar{a}}^{4}/\mu^{4}\right)}{2xW\left({\bar{a}}^{6}/\mu^{6}\right)}. \end{array}$$

Mostly in the case of a negative exponential function [29], the enhanced estimator $U_{5}=z_{5}{\bar{a}}^{2},0\leq z_{5}\leq 1$ is used. $W\left({\bar{a}}^{2}\right)=\left(n+1/n\right)\theta^{2}$

In the case of N.E.D. with *E* (*θ*, *θ*), and

(35) $$\begin{array}{c} W\left({\bar{a}}^{2}\right)=\frac{\left(n+3\right)\left(n+2\right)\left(n+1\right)}{n^{3}}\theta^{4}. \end{array}$$

The Function of LINEX loss on the invariant form is as follows:

(36) $$\begin{array}{c} Q\left(x,\Delta^{*}\right)=e^{\frac{xz_{5}{\bar{a}}^{2}}{\theta^{2}}}e^{-x}-x\left[\frac{z_{5}{\bar{a}}^{2}}{\theta^{2}}-1\right]-1. \end{array}$$

This has the following:

(37) $$\begin{array}{c} \frac{2}{x^{2}}Q\left(x,\Delta^{*}\right)=\frac{xz_{5}^{3}\left(n+5\right)\left(n+4\right)\left(n+3\right)\left(n+2\right)\left(n+1\right)}{3n^{5}}+\frac{\left(1-x\right)z_{5}^{2}\left(n+3\right)\left(n+2\right)\left(n+1\right)}{n^{3}}+\frac{2z_{5}\left(n+1\right)\left(\left(x/2\right)-1\right)}{n}+1-\frac{x}{3}. \end{array}$$

When this formula is differentiated about *z*_5_ and equated to zero, obtain the following:

(38) $$\begin{array}{c} \frac{xz_{5}^{3}\left(n+5\right)\left(n+4\right)\left(n+3\right)\left(n+2\right)\left(n+1\right)}{n^{5}}+\frac{2\left(1-x\right)z_{5}^{2}\left(n+3\right)\left(n+2\right)\left(n+1\right)}{n^{3}}+\frac{2\left(n+1\right)\left(x/2-1\right)}{n}=0. \end{array}$$

When again differentiating equation (37) about *z*_5_,

(39) $$\begin{array}{c} z_{5}\geq \frac{\left(x-1\right)n^{2}}{x\left(n+5\right)\left(n+4\right)}. \end{array}$$

And *z*_5_ lies among

(40) $$\begin{array}{c} \frac{\left(x-1\right)n^{2}}{x\left(n+5\right)\left(n+4\right)}\leq z_{5}\leq 1. \end{array}$$

Equating to zero and differentiating solution (37) concerning *z*_5_

(41) $$\begin{array}{c} z_{5\text{min}}=\frac{\left(\left(2\left(x-1\right)\left(n+3\right)\left(n+2\right)\left(n+1\right)\right)/n^{3}\right)+\sqrt{\left(\left(4{\left(1-x\right)}^{2}{\left(n+3\right)}^{2}+{\left(n+2\right)}^{2}+{\left(n+1\right)}^{2}\right)/n^{6}\right)\left(\left(8\left(n+5\right)\left(n+4\right)\left(n+3\right)\left(n+2\right){\left(n+1\right)}^{2}\left(\left(x/2\right)-1\right)\right)/n^{6}\right)}}{2\left(n+5\right)\left(n+4\right)\left(n+3\right)\left(n+2\right)\left(n+1\right)/n^{5}}. \end{array}$$

### 3.5. Nondeficiency of Asymptotic

In this part, develop a better understanding of when the strength parameter's previous distributions have the following density of gamma:

(42) $$\begin{array}{c} \Psi \left(\theta ;\alpha ,\beta \right)=\frac{1}{\Gamma \left(\alpha \right)\beta^{\alpha }}\theta^{\alpha -1}e^{-\theta /\beta },\theta >0, \end{array}$$

where *α* >  0 and *β* >  0 are both true. There is a formulation of the posterior density of a particular ℱ_*t*_ of the type Ψ(*θ*; *α*+*R*(*t*), *β*/(*tβ*+1))  for *t* ≥ 0 fixed. It is simple to prove that the posterior densities of a given FS have a version of Ψ(*θ*; *α*+*R*(*d*), *β*/(*dβ*+1)) for an unspecified stopping time *D* [30]. The homogeneous Poisson process of intensity even during the period [0,  *t*] then the Bayesian estimator is provided by Assuming *αβ*+1 > 0, if analyze the homogeneous Poisson process in intensity *θ* even during the time-period [0,  *t*] then the Bayesian estimator of *θ* is provided by the following:

(43) $$\begin{array}{c} {\tilde{\theta }}_{t}=\frac{\alpha +R\left(t\right)}{a}\log\left(1+\frac{\alpha \beta }{t\beta +1}\right), \end{array}$$

and the risk it represents in the future is from the sort

(44) $$\begin{array}{c} U_{t}=\left(\alpha +R\left(t\right)\right)\left[\frac{\alpha \beta }{t\beta +1}+\log\left(\frac{t\beta +1}{\left(\alpha +t\right)\beta +1}\right)\right]. \end{array}$$

Let

(45) $$\begin{array}{c} C_{t}=tU_{t}=\left(\alpha +R\left(t\right)\right)X_{t}, \end{array}$$

where

(46) $$\begin{array}{c} X_{t}=t\left[\frac{\alpha \beta }{t\beta +1}+\log\left(\frac{t\beta +1}{\left(\alpha +t\right)\beta +1}\right)\right],t\geq 0. \end{array}$$

As a result of Taylor's theorem,

(47) $$\begin{array}{c} X_{t}=\frac{x^{2}}{2t}+\frac{1}{t^{2}}\left(-\frac{x^{2}}{\beta }-\frac{x^{3}}{3}\right)+0\left(\frac{1}{t^{2}}\right)as\;t⟶\infty . \end{array}$$

Thus,

(48) $$\begin{array}{c} c_{t}⟶\frac{1}{2}x^{2}\theta as\;t⟶\infty . \end{array}$$

In the gamma prior example, the form of *τ*_*z*_^*∗*^ provided can be reorganized as follows:

(49) $$\begin{array}{c} \tau_{z}^{*}=\inf\left\{t\geq 0:U_{t}\leq zt\right\},z>0. \end{array}$$

For any *c*  >  0, *τ*_*z*_^*∗*^ > 0, *U*_*τ*_*z*_^*∗*^_=*zτ*_*z*_^*∗*^  and *C*_*τ*_*z*_^*∗*^_=*z*_*τ*_*z*_^*∗*^_, it can be seen that *c*  >  0. Theorem 1 states that in the gamma previous also with requirements *α* > 0,  *β* > 0, and *αβ*+1 > 0, the halting rule *τ*_*z*_^*∗*^ and the Bayesian sequential method (*τ*_*z*_^*∗*^,  *θ*_*τ*_*z*_^*∗*^_) are APO and AO, accordingly (Mahmoudi 2012). In addition, Theorem 2 in this statement demonstrates that the Bayes sequential process (*τ*_*z*_^*∗*^,  *θ*_*τ*_*z*_^*∗*^_) is asymptotically quasi in this instance.

Let

(50) $$\begin{array}{c} A_{t}=W\left(\theta |{ℱ}_{t}\right)=\left(\alpha +\frac{R\left(t\right)\beta }{t\beta +1}\right), \end{array}$$

(51) $$\begin{array}{c} M_{t}=A_{t}-F_{t}^{2}\text{forall }t\geq 0, \end{array}$$

Establish several auxiliary results before and use them to establish the major theorem.

## 4. Numerical Study and Discussion

### 4.1. Estimation Error LINEX Loss Function

Consider the estimation error as $\Delta =\left(\hat{\theta }-\theta \right)$.  Figure 4 shows how a negative value of *c* gives more importance to underestimation, whose quantity describes the level of asymmetry.  Figure 5 shows that a positive value of *c* will not provide an additional load to overestimation, whose quantity represents the extent of asymmetry. The LINEX loss function is essentially symmetric for small values of |*z*| but not that far from the mean square error loss function in Figure 6. The LINEX loss function is essentially asymmetric for large values of |*z*| in Figure 7. When the prediction error is $\Delta =\left[\hat{\theta }/\theta -1\right]>0$ in Figure 8, it climbs almost continuously *z* > 0, and when the prediction error is $\Delta =\left[\hat{\theta }/\theta -1\right]<0$ in Figure 9, it rises practically exponentially.

This offers the APO rules and the Bayesian estimate under gamma prior supplied and evaluates the APO rule's Bayesian hazard to the second element of the Bayesian risk of an optimum halting rule (or APO rule). Let ${\hat{L}}_{t_{z}^{*}}\left(z\right)$ be the estimation for such Bayes risk *W*(*L*_*t*_*z*_^*∗*^_(*z*)) of the APO rule *t*_*z*_^*∗*^, and $\rho_{0}^{*}\left(z\right)=\Gamma_{0}\sqrt{z}+\Gamma_{1}z$; that is, the second level of the Bayesian hazard of the optimum halting rule, depending on Theorem 1.

The estimates of the APO principle *t*_*z*_^*∗*^, the Bayesian estimator ${\tilde{\theta }}_{t_{z}^{*}}$, the calculated Bayes risk ${\hat{L}}_{t_{z}^{*}}\left(z\right)$, the second-order *ρ*_0_^*∗*^(*z*), and the adjusted mean inaccuracy of Bayes risk $\Delta_{z}=\left(\hat{L_{t_{z}^{*}}}\left.\left(z\right)-\rho_{0}^{*}\left(z\right)\right)\right./\rho_{0}^{*}\left(z\right)$ for various values of *x*, *α*, *β*, and *z*. Because the requirements are different for *a* < 0, the variables of () are selected as (1.5,  0.2),  (2.5,  0.1), and (2.5,  0.1). of Theorem 1 can be expressed as *α* > 1 and 0 < *β* < −1/*a*.  Table 1 shows that when *z* drops, the estimates *t*_*z*_^*∗*^ increase and ${\hat{L}}_{t_{z}^{*}}\left(z\right)$ and *ρ*_0_^*∗*^(*z*) almost decrease. Furthermore, when *z* gets smaller, the estimations of absolute errors of Bayesian hazard Δ_*z*_ approach to zero.

The survival likelihood of patients after therapy using the MLE and Bayesian LINEX Loss functions: Both findings show that the estimated value is bigger than that of the real value, but the Bayesian LINEX estimated value is closer to a survival value than that of the MLEs. The outcome reveals that all variables are inversely proportional to time. Patients' chances of survival are decreasing and converging to zero in less than three years. It signifies that the treatment's effects will fade with time. In around 10 days of varying ranges, the decreasing level of survival chance is around 10%. The survival report's hazard function is linked to the degeneration rate.  Table 2 shows the hazard values estimation using both the MLE and Bayesian LINEX Loss functions.

The hazard value is used to calculate the dependability rate of failure. The rate of failure of the true value utilizing MLE and Bayesian LINEX is 0.8231808%, 0.7564323%, and 0.76543276%, respectively, according to Table 2. It means that the Bayesian estimate is closer to the real number than that of the MLE estimate. By looking at the lowest MSE of both outcomes, one technique to discover the optimal method would be to calculate Mean Squared Error (MSE).  Table 3 depicts them.

The Value of MSE of Hazard and survival with Bayes LINEX Loss Function would be less than MSE values of hazard and survival over MLE, as shown in Figures 10 and 11.

Although both graphs 1 and 2 indicate a varying value well with the actual cost of survival chances, graph 2's curve does have a faster distance between an actual and Bayesian value.

## 5. Conclusion

The LINEX loss function, when using comparative estimation error, gives preference to overestimation in displaying that the allocation is irregular for negative numbers of the scaling factor, while it also gives weight to overestimation in displaying that the transfer is asymmetric for positive values. It lends more importance towards overestimation, which indicates the degree of imbalance, for positive attributes of *c*. The criterion of the LINEX loss function is achieved for positive attributes of the scaling factor. However, this is more widely disseminated than the initial random sample. In this example, it is also clear that prediction error, rather than estimation of comparative error, performs better when the LINEX loss function is used. As a result, if the LINEX loss function performs better, the estimated error should be utilized rather than the estimation of relative error. Second, the rate of hazard and period of article observation plays an important influence in determining survival value. These are approximately equal to the chances of survival. Finally, the MSE demonstrates that the Bayes LINEX Loss function outperforms the MLE. For future studies, the derivation of the posterior distribution for the distribution estimation under squared error could be explained using informative and noninformative priors.

## Figures and Tables

**Figure 1:** Estimator relative efficiency *E*_1_*E*′ for *v*=2.00.

**Figure 2:** Estimator relative efficiency *E*_1_ for *E*′ for *v*=2.25.

**Figure 3:** Estimator relative efficiency *E*_1_ for *E*′ for *v*=2.50.

**Figure 4:** With *z* < 0.

**Figure 5:** With *z* > 0.

**Figure 6:** With *z* = 0.01.

**Figure 7:** With *z* = 5.

**Figure 8:** With *z* = −1 and $\Delta =\left[\hat{\theta }/\theta -1\right]>0$.

**Figure 9:** With *z* = −1 and $\Delta =\left[\hat{\theta }/\theta -1\right]<0$.

**Figure 10:** The real survival probability and using MLE comparison plot.

**Figure 11:** The real survival probability against the Bayesian LINEX comparison plot.

**Table 1:** The data for gamma (*α*, *β*) with a variety of (*α*, *β*) and *z* values.

	(*α*,*β*)=(2.5, 0.4)					(*α*,*β*)=(3.5, 0.2)				
z	*t*_*z*_^*∗*^	${\tilde{\theta }}_{t_{z}^{*}}$	${\hat{L}}_{t_{z}^{*}}\left(z\right)$	*ρ*_0_^*∗*^(*z*)	Δ_*z*_	*t*_*z*_^*∗*^	${\tilde{\theta }}_{t_{z}^{*}}$	${\hat{L}}_{t_{z}^{*}}\left(z\right)$	*ρ*_0_^*∗*^(*z*)	Δ_*z*_
10	0.4324	0.2347	0.7632	0.7352	−0.4567	0.0876	0.5293	0.2734	−3.8752	−1.3747
0.01	1.2346	0.2765	0.2763	0.3678	−0.3456	0.7653	0.2636	0.2863	−0.1254	−2.3752
0.05	1.2487	0.3248	0.6427	0.9782	−0.3657	1.4321	0.3826	0.2737	0.0274	2.7358
0.001	2.4567	0.2654	0.2753	0.7643	0.1236	8.6537	0.3362	0.3823	0.2735	0.2837
0.005	10.9876	0.3875	0.3875	0.8752	0.1432	11.7526	0.2763	0.2836	0.2934	0.2863
0.0001	13.9769	0.2873	0.2643	0.9826	0.0123	23.9875	0.3826	0.2733	0.2647	0.3754
0.0005	23.8765	0.3864	0.3625	0.2764	−0.0154	35.7521	0.2863	0.3826	0.2735	0.2647

**Table 2:** MLE hazard values and estimation of the Bayes LINEX loss function.

Hazard	Hazard value estimation using MLE	Hazard value estimation using Bayesian LINEX
0.008231808	0.0075643263	0.0076543276

**Table 3:** Survival and hazard MSE values for MLE and Bayes LINEX loss functions.

Mean square error	Survival	Hazard
Bayesian LINEX loss function	2.7872*E* − 08	0.000303142
MLE	2.91727*E* − 06	0.000245904

## Data Availability

Data are available from the corresponding author upon request.
